RETRACTED

# Gadd153 and NF-κB Crosstalk Regulates 27-Hydroxycholesterol-Induced Increase in BACE1 and β-Amyloid Production in Human Neuroblastoma SH-SY5Y Cells

**DOI:** 10.1371/journal.pone.0070773

**Published:** 2013-08-09

**Authors:** Gurdeep Marwarha, Shaneabbas Raza, Jaya R. P. Prasanthi, Othman Ghribi

**Affiliations:** Department of Pharmacology, Physiology and Therapeutics, University of North Dakota School of Medicine and Health Sciences, Grand Forks, North Dakota, United States of America; National Institute of Health, United States of America

## Abstract

β-amyloid (Aβ) peptide, accumulation of which is a culprit for Alzheimer’s disease (AD), is derived from the initial cleavage of amyloid precursor protein by the aspartyl protease BACE1. Identification of cellular mechanisms that regulate BACE1 production is of high relevance to the search for potential disease-modifying therapies that inhibit BACE1 to reduce Aβ accumulation and AD progression. In the present study, we show that the cholesterol oxidation product 27-hydroxycholesterol (27-OHC) increases BACE1 and Aβ levels in human neuroblastoma SH-SY5Y cells. This increase in BACE1 involves a crosstalk between the two transcription factors NF-κB and the endoplasmic reticulum stress marker, the growth arrest and DNA damage induced gene-153 (gadd153, also called CHOP). We specifically show that 27-OHC induces a substantial increase in NF-κB binding to the BACE1 promoter and subsequent increase in BACE1 transcription and Aβ production. The NF-κB inhibitor, sc514, significantly attenuated the 27-OHC-induced increase in NF-κB-mediated BACE1 expression and Aβ genesis. We further show that the 27-OHC-induced NF-κB activation and increased NF-κB-mediated BACE1 expression is contingent on the increased activation of gadd153. Silencing gadd153 expression with siRNA alleviated the 27-OHC-induced increase in NF-κB activation, NF-κB binding to the BACE1 promoter, and subsequent increase in BACE1 transcription and Aβ production. We also show that increased levels of BACE1 in the triple transgenic mouse model for AD is preceded by gadd153 and NF-κB activation. In summary, our study demonstrates that gadd153 and NF-κB work in concert to regulate BACE1 expression. Agents that inhibit gadd153 activation and subsequent interaction with NF-κB might be promising targets to reduce BACE1 and Aβ overproduction and may ultimately serve as disease-modifying treatments for AD.

## Introduction

Alzheimer Disease (AD) is the most common neurodegenerative disorder and the fifth leading cause of death in the elderly. Extracellular deposition of aggregated Amyloid-β (Aβ) peptide in *senile plaques* and intraneuronal accumulation of aggregated hyperphosphorylated microtubule-associated protein tau (τ) in *neurofibrillary tangles* (NFT) are the two major pathological hallmarks of AD. The etiology of AD is unknown, but it is widely accepted that increased production and accumulation of Aβ is an instigator of the neurodegenerative processes observed in AD [1]. Reduction in Aβ production and accumulation is an appealing strategy to reduce the progression of AD. Aβ is derived from the amyloid precursor protein (APP) through an initial cleavage by aspartyl protease BACE1 and subsequent cleavage by the γ-secretase enzyme complex [2], [3]. The initial cleavage of APP by BACE1 is the rate-limiting step in Aβ production [2], [3]. Several studies have shown that BACE1 protein, mRNA, and activity are upregulated in AD brains [4]–[7].

RETRACTED

Stress in endoplasmic reticulum (ER) may play a role in the pathophysiology of many diseases including AD [8]–[10]. Sustained ER stress upregulates the gene expression of several deleterious transcription factors including that of the growth arrest and DNA damage-induced gene153 (gadd153; also known as C/EBP homologous protein, CHOP). Interestingly, gadd153 has been shown to enhance NF-κB signaling [11], suggesting that gadd153 can crosstalk with NF-κB, and that NF-κB activation can be a downstream event to activated gadd153. Multiple lines of evidence suggest that, in addition to being an important regulator of inflammation, NF-κB also regulates the transcription of BACE1, as evidenced by the presence of κB sites in the BACE1 promoter region [12]–[14]. More evidence of the tight link of NF-κB to the pathophysiology of AD is the observation that this transcription factor is activated in AD patients [12], [13], [15].

Our published studies demonstrated that the cholesterol oxidized metabolite (oxysterol) 27-hydroxycholesterol (27-OHC) increases BACE1 levels in hippocampal organotypic slices from adult rabbits [16] and in human SH-SY5Y neuroblastoma cells [17]. The oxysterol 27-OHC has been shown to accumulate in AD brains [18]. We also showed that 27-OHC induced ER-mediated gadd153 and NF-κB activation in ARPE cells [19] and SH-SY5Y cells [20]. We propose that, because gadd153 and NF-κB may work in concert to upregulate BACE1, a crosstalk between gadd153 and NF-κB would enhance Aβ production and accumulation, and may thus increase the risk for AD. Inhibition of gadd153 would therefore reduce NF-κB and BACE1 expression, prevent Aβ accumulation, and may have a translation potential for reducing the propgression of AD. In the present study, we not only demonstrate the involvement of NF-κB in 27-OHC-induced increase in BACE1 expression levels, but also establish the dynamic interplay between gadd153 and NF-κB in the regulation of BACE1 expression in response to treatment with the oxysterol 27-OHC.

RETRACTED

## Methods

### Reagents

27-OHC was purchased from Medical Isotopes (Pelham, NH), the NF-κB inhibitor sc514 from Tocris Bioscience (Ellisville, MO), the reporter constructs encoding NF-κB response elements conjugated to the firefly luciferase gene from SA Biosciences (Frederick, MD), and the human BACE1 promoter construct conjugated to the firefly luciferase gene was purchased from SwitchGear Genomics (Menlo Park, CA). All cell culture reagents, with the exception of fetal bovine serum (Atlanta Biologicals, Lawrenceville, GA) and antibiotic/antimycotic mix (Sigma Aldrich, Saint Louis, MO) were from Invitrogen (Carlsbad, CA). Human SH-SY5Y neuroblastoma cells were purchased from ATCC (Manassas, VA).

### Cell Culture and Treatments

Human neuroblastoma SH-SY5Y cells were grown in DMEM/F12 medium containing 10% fetal bovine serum (FBS) and 1% antibiotic/antimycotic mix. Cells were maintained at 37°C in a saturated humidity atmosphere containing 95% air and 5% CO_2_. After reaching 80% confluence, cells were incubated for 24 hours at 37°C in cell medium with vehicle, 5 µM 27-OHC, 5 µM NF-κB inhibitor sc514, or 5 µM 27-OHC +5 µM sc514. siRNA for gadd153 and the respective scrambled non-silencing control siRNA were purchased from Santa Cruz Biotechnology (Santa Cruz, CA). The following human gadd153 double-stranded siRNA sequences (5′ → 3′ orientation) were used (A): Sense GAAGGCUUGGAGUAGACAAtt, Antisense UUGUCUACUCCAAGCCUUCtt; (B): Sense GGAAAGGUCUCAGCUUGUAtt, Antisense UACAAGCUGAGACCUUUCCtt; (C): Sense GUCUCAGCUUGUAUAUAGAtt, Antisense UCUAUAUACAAGCUGAGACtt. The transfection of siRNA was performed in the cells with siRNA transfection reagent (Santa Cruz Biotechnology) and siRNA transfection medium (Santa Cruz Biotechnology) according to the manufacturer’s recommendation. The siRNAs stock solution (10 µM) was prepared by dissolving 3 nmol of siRNAs in 330 µL of RNAse free water and further diluted 1∶50 using transfection reagent and transfection medium following manufacturer’s protocol to yield a final concentration of 200 nM. The cells were transfected for 16 hours followed by 24 hour incubation in normal media before being subjected to respective treatments.

### Animal Study

The precise role of gadd153 in AD and the extent to which gadd153 is activated in AD are ill-defined. In order to determine whether gadd153 and NF-κB are activated in transgenic mice model for AD, we used 3, 6 and 12 month-old male triple transgenic (3xTg-AD) mice (n = 6 per group). The 3xTg-AD mouse model harbors 3 mutant genes, namely amyloid- β protein precursor (AβPPswe), presenilin-1 (PS1M146 V) and tau (P301 L). The 3xTg-AD mice used in the present study are from a colony maintained for more than 7 generations in our facility. Our mice colony was developed from 3xTg-AD mice obtained from Dr. Frederic Calon, Laval University [21], [22]. Dr. Calon’s colony, maintained on a C57BL/6J background for more than 10 generations in his facility, was originally derived from a colony generated from homozygous founders obtained from Dr. Frank LaFerla on a C57BL/6J x129SVJ background [23]. Mice were deeply anesthetized and perfused trans-cardially with phosphate-buffered saline (PBS). Brains were promptly removed and processed for Western blot analyses.

RETRACTED

### Ethics Statement

All animal procedures were carried out in accordance with the U.S. Public Health Service Policy on the Humane Care and Use of Laboratory Animals and were approved by the Institutional Animal Care and Use Committee at the University of North Dakota (Protocol 110.3-3).

### Western Blot Analysis

Treated SH-SY5Y cells were washed with PBS and trypsinized to collect the cells and centrifuged at 5000 g. The pellet was washed again with PBS and homogenized in NE-PER tissue protein extraction reagent (Thermo Scientific, Rockford, IL) supplemented with protease and phosphatase inhibitors. Hippocampi isolated from 3XTg-AD and non-transgenic control mice brains were homogenized in T-PER tissue protein extraction reagent (Thermo Scientific) also containing protease and phosphatase inhibitors. Total, cytosolic, or nuclear proteins (10 µg) were separated on SDS-PAGE gels, transferred to a polyvinylidene difluoride membrane (BioRad, Hercules, CA), and incubated with the following monoclonal antibodies to : gadd153 (1∶100, Abcam, Cambridge, MA), BACE1 (1∶1000; Millipore, Bedford, MA), p65 mouse antibody (1∶200; Cell Signaling, Boston, MA), p50 (1∶200; Cell Signaling, Boston, MA), IKKα (1∶500; Cell Signaling, Boston, MA), anti-IKKβ (1∶500; Cell Signaling, Boston, MA), p-Ser^176/180^ IKKα/β (1∶500; Cell Signaling, Boston, MA), anti-IKBα (1∶2000, Abcam), and anti p- Ser^32^ IKBα (1∶200, Santa Cruz). β-actin and Lamin A/C were used as a gel loading control for cytosolic homogenates and nuclear homogenates respectively. The blots were developed with enhanced chemiluminescence (Immun-star HRP chemiluminescent kit, Bio-Rad, Hercules, CA). Bands were visualized on a polyvinylidene difluoride membrane and analyzed by LabWorks 4.5 software on a UVP Bioimaging System (Upland, CA). Quantification of results was performed by densitometry and the results analyzed as total integrated densitometric values (arbitrary units).

### Quantitative Real Time RT-PCR Analysis

Total RNA was isolated and extracted from treated cells using the 5 prime “PerfectPure RNA tissue kit” (5 Prime, Inc., Gaithersburg, MD). RNA estimation was performed using “Quant-iT RNA Assay Kit” and a Qubit fluorometer according to the manufacturer’s protocol (Invitrogen, Carlsbad, CA). cDNA was synthesized by reverse transcribing 1 µg of extracted RNA using an iScript cDNA synthesis kit” (BioRad, Hercules, CA). The oligomeric primers (Sigma, St Louis, MO) used to amplify BACE1 mRNA are enumerated in Table 1. The cDNA amplification was performed using an iQ SYBR Green Supermix kit following the manufacturer’s instructions (BioRad, Hercules, CA). The amplification was performed using an iCycler iQ Multicolor Real Time PCR Detection System (BioRad, Hercules, CA). The expressions of specific BACE1 transcripts amplified were normalized to the expression of glyceraldehyde -3-phosphate dehydrogenase (GAPDH).

RETRACTED

**Table 1:** Primers designed and used for RT-PCR, EMSA, and ChIP analyses.

Gene	Primer	Gene Bank Accession Number	Sequence	Assay
BACE1	Forward	NM 012104	5′-aggttaccttggcgtgtgtc-3′	RT-PCR
BACE1	Reverse	NM 012104	5′-gaggcaatctttgcaccaat-3′	RT-PCR
BACE1		NT 033899	5′-ggctaacatggtgaattcccgtctccacta-3′	EMSA
BACE1	Forward	NT 033899	5′-tgaggcaggcagataacttg-3′	ChIP
BACE1	Reverse	NT 033899	5′-gcctcctcaagcgattctc-3′	ChIP

### ELISA Immunoassay

Aβ40 and Aβ42 levels were quantified in the media (secreted) and cellular homogenates (intracellular) using an ELISA immunoassay kit (Invitrogen, Carlsbad, CA) as per the manufacturer’s protocol. Following treatments, the culture medium was collected, supplemented with protease and phosphatase inhibitors cocktail, and centrifuged at 16,000 *g* for 5 min at 4°C. 100 µl of supernatant was used for the quantification of secreted Aβ40 and Aβ42 levels by colorimetric sandwich ELISA according to the manufacturer’s protocol. To measure the levels of intracellular Aβ40 and Aβ42 in the cellular homogenates, cells were trypsinized and collected by centrifugation at 5000 g and the cell pellet (∼100 mg) was homogenized thoroughly with 8x mass of cold 5 M guanidine Hcl/50 mM Tris–HCl. The homogenates were mixed for 3–4 h at room temperature. The samples were diluted with cold reaction buffer (Dulbecco’s phosphate-buffered saline with 5% BSA and 0.03% Tween-20 supplemented with 1x protease inhibitor cocktail) and centrifuged at 16,000 *g* for 20 min at 4°C. The supernatant was decanted, diluted at 1∶1 with standard diluent buffer, and quantified by colorimetric sandwich ELISA kits. Intracellular Aβ levels in the cellular homogenates were normalized to total protein content in the samples. Treatments were performed in quadruplet, and the quantity of Aβ in each sample was measured in duplicate. The secreted Aβ40 and Aβ42 levels measured in the culture medium are expressed in pg/mL of media.

RETRACTED

### Electrophoretic Mobility Shift Assay (EMSA)

The Electrophoretic Mobility Shift Assay (EMSA) was performed using a kit from Active Motif (Carlsbad, CA) following manufacturer’s protocol. Nuclear extract was prepared using NE-PER protein extraction reagent following the manufacturer’s instructions (Thermo Scientific, Rockford, IL). The human BACE1 promoter region spanning 5000 nucleotides upstream of the transcription initiation site in BACE1 gene was scanned for NF-κB binding consensus sequences using the “TFsearch” online program that searches highly correlated sequence fragments against TFMATRIX transcription factor binding site profile database in ‘TRANSFAC’ databases. The human BACE1 promoter contains a NF-κB consensus motif 2549 nucleotides upstream of the transcription start site. The 5′-biotin labeled and unlabeled oligonucleotide probes that correspond to the NF-κB binding site in the human BACE1 promoter region (−2559 to −2530 of the BACE1 promoter) (Table 1) were purchased from Sigma Aldrich (St Louis, MO). 10 µg of nuclear proteins were incubated with either 20 femto moles of biotin labeled oligonucleotide probe or 4 pico moles of unlabelled oligonucleotide. To exhibit specificity of the oligonucleotide probes, unlabelled oligonucleotide probe was used as a specific competitor for binding reactions at a concentration of 200 fold of the concentration of the biotin labeled probe. 1 µg of Poly d(I–C) was used as a non-specific competitor for binding reactions. The resulting binding reaction mix was loaded and resolved on a 5% TBE gel (BioRad, Hercules, CA) followed by transfer onto a nylon membrane. The bands were visualized using the HRP-Streptavidin – Chemiluminescent reaction mix provided with the kit on a UVP Bioimaging System (Upland, CA).

### Chromatin Immunoprecipitation (ChIP) Analysis

ChIP analysis was performed to evaluate the extent of NF-κB binding to the DNA elements in the BACE1 promoter regions respectively using “SimpleChIP™ Enzymatic Chromatic IP kit” from Cell Signaling (Boston, MA). Briefly, cells from each treatment group (3×10^6^ cells) were washed with PBS, trypsinized, centrifuged at 5000 g. The pellet containing the cells was further washed with PBS and cross-linked using 37% formaldehyde for 15 min followed by the addition of glycine solution to cease the cross-linking reaction. The cells were washed with 4x volumes of 1x PBS and centrifuged at ∼220 g for 5 min. The pellet was resuspended and incubated for 10 min in 5 ml of tissue lysis buffer containing DTT and protease and phosphatase inhibitors. The subsequent steps to isolate the cross-linked chromatin were performed according to the manufacturer’s protocol. The cross-linked chromatin from each sample was apportioned into three equal parts. One third of the cross-linked chromatin was set aside as “input”. One third of the cross-linked chromatin from each sample was incubated with 5 µg of p65 mouse antibody (Abcam, Cambridge, MA), while the remaining one third of the cross-linked chromatin from each sample was incubated with 5 µg of normal Rabbit IgG to serve as negative control. The cross-linked chromatin samples were incubated overnight at 4°C with their respective antibodies. The DNA-protein complexes were collected with Protein G agarose beads and washed to remove non-specific antibody binding. The DNA from the DNA-protein complexes from all the samples including the input and negative control was reverse cross-linked by incubation with 2 µL of Proteinase K for 2 hours at 65°C. The crude DNA extract was eluted and then washed several times with wash buffer containing ethanol (provided with the kit) followed by purification with the use of DNA spin columns provided by the manufacturer. The pure DNA was eluted out of the DNA spin columns using 50 µL of the DNA elution buffer provided in the kit. 1 µL of the purified DNA was used for DNA concentration analysis using the “Quant-iT™ dsDNA Assay kit from Invitrogen (Carlsbad, CA) The DNA fragment size was determined by electrophoresis on a 1.2% agarose FlashGel^R^ system (Lonza, Rockland, ME). The relative abundance of the p65 antibody precipitated chromatin containing the NF-κB binding site in the BACE1 promoter region was determined by qPCR using an iQ SYBR Green Supermix kit following the manufacturer’s instructions (BioRad, Hercules, CA) and sequence specific primers (Table 1). The amplification was performed using an iCycler iQ Multicolor Real Time PCR Detection System (BioRad, Hercules, CA).The fold enrichment was calculated using the ΔΔC_t_ method (Livak & Schmittgen, 2001) which normalizes ChIP C_t_ values of each sample to the % input and background.

RETRACTED

### Luciferase Reporter Assays

Constructs encoding NF-κB response element and human BACE1 promoter conjugated to the firefly luciferase gene were used in the study. SH-SY5Y cells were plated in 96-well plates at a density of 2×10^4^cells/well. The cells were transfected when 80% confluent with 0.25 µg of reporter constructs. Respective non-inducible reporter constructs containing constitutively expressing *Renilla* luciferase were used as negative internal controls. Constitutively expressing GFP constructs were used as positive control to determine transfection efficiency. Cells were incubated for 24 hours with Opti-MEM serum free medium (Invitrogen, Carlsbad, CA) containing the reporter constructs dissolved in transfection reagent. After 24 hours the medium was changed and the cells were incubated in normal DMEM/F12 medium containing 10% FBS and cells were treated with the different treatment regimens. The cells were treated in triplicate and harvested 24 hours later and subjected to dual-luciferases assay. The dual-luciferase assay was performed using a “Dual-Luciferase Reporter Assay System” (Promega, Madison, WI). The luminescence recorded is expressed as Relative Luminescence Units (RLU) and normalized to per mg protein. Unit value was assigned to control and the magnitude of differences among the samples is expressed relative to the unit value of control cells.

### Statistical Analysis

The significance of differences among the samples was assessed by One Way Analysis of Variance (One Way ANOVA) followed by Tukey’s post-hoc test. Statistical analysis was performed with GraphPad Prism software 4.01. Quantitative data for Western blotting analysis are presented as mean values ± S.E.M with unit value assigned to control and the magnitude of differences among the samples being expressed relative to the unit value of control. Quantitative data for RT-PCR analysis are presented as mean values ± S.E.M, with reported values being the product of absolute value of the ratio of BACE1 to GAPDH mRNA multiplied by 1000000.

## Results

### 27-OHC Increases BACE1 Expression and Subsequent Aβ Production by Activating NF-κB Signaling

NF-κB family of proteins exist as homodimers or heterodimers of five different proteins or subunits, namely – p65 (RelA), RelB, c-Rel, p50, and p52. Among the 15 known heterodimers and homodimers that exist, the p65-p50 heterodimeric NF-κB complex is the most common and well-studied [24]. In resting cells, NF-κB heterodimers are sequestered in the cytosol through interaction with IκB proteins which results in inhibition of NF-κB nuclear translocation and subsequent DNA binding and transcriptional activation [25]. Stimulus specific activation of IκB kinases (IKKs) leads to phosphorylation, ubiquitination and proteasomal degradation of IκB proteins thereby releasing and allowing the nuclear translocation of the free NF-κB dimer [24], [26]. We therefore determined the p65 and p50 nuclear levels in cells treated with 27-OHC as a surrogate marker of NF-κB activation. 27-OHC treatment elicited a 2.2-fold increase in p65 and a 2-fold increase in p50 translocation to the nucleus (Fig. 1a,b). We also determined the involvement of NF-κB in 27-OHC-induced increase in BACE1 expression. To this end, we treated SH-SY5Y cells with 27-OHC in the presence and absence of sc514, a selective IKKβ (IκB kinase β) inhibitor that inhibits IκB phosphorylation, subsequent ubiquitination and degradation thereby keeping NF-κB sequestered in the cytosol and inhibiting NF-κB signaling [25]. sc514 inhibits IKKβ with an IC_50_ of 3–12 µM [27]. We found that, while 27-OHC induces ∼2-fold increase in BACE1 protein levels (Fig. 1c,d) and 3.5-fold increase in BACE1 mRNA expression (Fig. 1e), treatment with the NF-κB inhibitor substantially reduced the 27-OHC-induced increase in BACE1 expression levels. Additionally, the NF-κB inhibitor did not elicit any significant effects on the basal expression levels of BACE1 (Fig. 1c–e). We next determined, the binding of NF-κB to the BACE1 promoter region using ChIP analysis and BACE1 promoter activity assay using a BACE1 promoter construct. We found that 27-OHC induces a substantial increase in NF-κB binding to the BACE1 promoter (Fig. 1f). To further demonstrate that the changes in NF-κB binding to the BACE1 promoter result in changes in transcription of BACE1, we performed NF-κB reporter activity assay and BACE1 promoter analysis using a dual-luciferase assay system. Dual-luciferase assay shows that 27-OHC elicited a 4-fold increase in NF-κB reporter activity (Fig. 1g). Furthermore, 27-OHC also increased the BACE1 promoter activity by ∼4.5-fold as determined by a dual-luciferase assay analysis (Fig. 1h). Importantly, the NF-κB inhibitor significantly attenuated the NF-κB binding to the BACE1 promoter region by ∼50% in absence or presence of 27-OHC as demonstrated by ChIP analysis (Fig. 1f). Treatment with sc514 also reduced the 27-OHC-induced increase in BACE1 promoter activity by ∼60% as demonstrated by dual luciferase assay (Fig. 1h). This suggests that activation of the transcription factor NF-κB predominantly mediates the 27-OHC-induced increase in BACE1 expression. However, the NF-κB inhibitor did not affect the basal BACE1 promoter activity (Fig. 1h) despite evoking a substantial reduction in the basal binding of NF-κB to the BACE1 promoter (Fig. 1f).

RETRACTED

**Figure 1:** 27-OHC induces NF-κB activation and subsequently increases NF-κB-mediated BACE1 expression. (a,b) 27-OHC significantly increases the levels of the p65 and the p50 subunits of the NF-κB in the nuclear homogenates, and (c–e) increases the protein and mRNA levels of BACE1; treatment with the NF-κB inhibitor sc514 attenuates the 27-OHC-induced increase in protein and mRNA expression of BACE1. (f) ChIP analysis shows that 27-OHC increases the binding of NF-κB in the BACE1 promoter region. (g) Dual luciferase assay demonstrates that 27-OHC increases the NF-κB transcriptional activity as measured by a significant increase in NF-κB reporter activity. (h) Dual luciferase assay demonstrates that 27-OHC significantly increases the BACE1 promoter activity, while the NF-κB inhibitor sc514 decreases the 27-OHC-induced increase in BACE1 promoter activity. Data is expressed as Mean+S.E.M and includes determinations made in four separate cell culture experiments (n = 4). *p<0.05, **p<0.01, and ***p<0.001 versus control, ^†^ p<0.05, ^††^ p<0.01, and ^†††^ p<0.001 versus 27-OHC.

The cleavage of Amyloid-β Precursor Protein (APP) by BACE1 is the rate limiting step in Aβ production. We determined the impact of inhibition of NF-κB activation and signaling on basal as well as 27-OHC-induced increase in Aβ levels. Consistent with our previously published studies [16], [17], 27-OHC evoked ∼2-fold increase in intracellular Aβ42 and a ∼1.7-fold increase in levels intracellular Aβ40 levels as determined by ELISA immunoassay (Fig. 2a,b). Treatment with 27-OHC also elicited a ∼2.2-fold increase in Aβ42 and a ∼1.7-fold increase in Aβ40 secreted in the media (Fig. 2c,d). However in the presence of the NF-κB inhibitor sc514, 27-OHC elicited only a ∼1.4-fold increase in intracellular Aβ42 and no significant increase in intracellular Aβ40 levels compared to basal levels (Fig. 2a,b). Furthermore, the NF-κB inhibitor sc514 also significantly attenuated the 27-OHC-induced increase in secreted Aβ42 by ∼33% and completely reversed the 27-OHC-induced increase in secreted Aβ40. This further suggests that NF-κB plays an indispensable role in 27-OHC-induced increase in BACE1 expression levels and subsequent increase in Aβ levels. However, consistent with the lack of effect of the NF-κB inhibitor on the basal expression levels of BACE1 (Fig. 1d,e) and BACE1 promoter activity (Fig. 1h), the NF-κB inhibitor sc514 did not elicit any effect on the basal levels of Aβ42 (intracellular and secreted) and Aβ42 (intracellular and secreted) (Fig. 2a–d).

**Figure 2:** 27-OHC-induced increase in the levels of intracellular as well as secreted forms of Aβ42 and Aβ40 is contingent on NF-κB activation. (a–d) ELISA immunoassay demonstrates that 27-OHC increases the levels of intracellular and secreted Aβ42 and Aβ40, while the NF-κB inhibitor sc514 mitigates the 27-OHC-induced increase in both intracellular and secreted Aβ42 and Aβ40. Data is expressed as Mean+S.E.M and includes determinations made in four separate cell culture experiments (n = 4). *p<0.05, **p<0.01, and ***p<0.001 versus control, ^††^ p<0.01 and ^†††^ p<0.001 versus 27-OHC.

### 27-OHC Increases NF-κB Activation by Evoking ER Stress and Inducing gadd153 Expression

Western blot analyses shows that siRNA to gadd153 efficiently reduces gadd153 levels in cells treated with 27-OHC (Fig. 3a). We determined whether gadd153 expression is required for NF-κB activation. To this end, we determined NF-κB activation and nuclear translocation by determining the nuclear levels of p65 and p50 subunits of the NF-κB heterodimeric complex in response to 27-OHC treatment in both the native and gadd153-silenced SH-SY5Y cells. 27-OHC evoked a 2-fold increase in p65 and a 2.5-fold increase in p50 translocation to the nucleus in cells untreated with siRNA to gadd153 (3b–d). However, 27-OHC treatment s did not elicit significant increase in p65 and p50 levels in the nucleus of gadd153-silenced SH-SY5Y cells (Fig. 3b–d). This suggests that 27-OHC induces NF-κB activation and its subsequent nuclear translocation by evoking ER stress-induced increase in gadd153 expression.

RETRACTED

**Figure 3:** 27-OHC-induced nuclear translocation of NF-κB is contingent on gadd153 activation. (a) siRNA to gadd153 suppresses the 27-OHC-induced increase in gadd153 protein levels. (b–d) siRNA to gadd153 attenuates the 27-OHC-induced increase in p65 and p50 subunit translocation to the nucleus. Data is expressed as Mean+S.E.M and includes determinations made in four separate cell culture experiments (n = 4). ***p<0.001 versus control, ^††^ p<0.01 and ^†††^ p<0.001 versus 27-OHC.

### 27-OHC Fails to Increase NF-κB-mediated BACE1 Expression and Aβ Production in gadd153 Silenced Cells

As we found that gadd153 is required for 27-OHC-induced NF-κB activation, and given that NF-κB increases BACE1 expression levels, we determined the involvement of gadd153 in 27-OHC-induced increase in BACE1 expression. To this end, we silenced gadd153 gene expression with siRNA in SH-SY5Y cells prior to treatment with 27-OHC. Treatment with 27-OHC elicited only a 1.3-fold increase in BACE1 protein levels and a 1.5-fold increase in BACE1 mRNA in gadd153 silenced cells compared to a ∼2.1-fold and ∼3-fold increase in BACE1 protein and mRNA levels respectively in native SH-SY5Y cells (Fig. 4a–c). However, the silencing of gadd153 expression did not elicit any effect on the basal expression levels of BACE1 (Fig. 4a–c). To correlate the decreased nuclear translocation of NF-κB in gadd153-silenced cells with the decreased expression levels of BACE1, we performed EMSA and ChIP analysis to determine the binding of NF-κB to the BACE1 promoter region in gadd153-silenced cells. Silencing gadd153 expression resulted in a significant reduction in the 27-OHC-induced increase in NF-κB binding to the exogenous DNA sequence that corresponds to the NF-κB-binding site in the BACE1 promoter as determined by EMSA (Fig. 4d). ChIP analysis also corroborated the EMSA data and revealed an ∼47% reduction in the NF-κB binding to the BACE1 promoter in gadd153-silenced cells treated with the 27-OHC compared 27-OHC-treated native cells. Gadd153-silenced cells treated with 27-OHC elicited a ∼4.5-fold increase in NF-κB binding to the BACE1 promoter compared to a ∼8.5-fold increase in NF-κB binding to the BACE1 promoter in 27-OHC-treated native cells (Fig. 4e).

RETRACTED

**Figure 4:** 27-OHC-induced NF-κB-mediated increase in BACE1 transcription and expression is contingent on gadd153 expression. (a–c) siRNA to gadd153 mitigates the 27-OHC-induced increase in BACE1 protein levels and mRNA expression. (d) EMSA shows that 27-OHC increases the binding of NF-κB to the exogenous DNA sequence that corresponds to the NF-κB binding site in the BACE1 promoter; silencing gadd153 expression reduces the increase in the binding of NF-κB. (e) ChIP analysis shows that siRNA to gadd153 decreases the 27-OHC-induced increase in binding of NF-κB to the BACE1 promoter. (f,g) Dual luciferase assay demonstrates that siRNA to gadd153 decreases the 27-OHC-induced increase in NF-κB transcriptional activity and BACE1 promoter activity. (h) Levels of gadd153 are detectable in hippocampus of 3, 6, and 12 month-old 3xTg-AD, while NF-κB levels are detectable in hippocampus of 6 and 12month-old, and BACE1 levels increasing only in 12 month-old 3xTg-AD. Data in a-g is expressed as Mean+S.E.M and includes determinations made in four separate cell culture experiments (n = 4). *p<0.05, **p<0.01, and ***p<0.001 versus control, ^††^ p<0.01 and ^†††^ p<0.001 versus 27-OHC.

To implicate gadd153 as the mediator of 27-OHC-induced increase in NF-κB-targeted BACE1 expression, we next performed dual-luciferase analysis to determine the extent of NF-κB transcriptional activity and BACE1 promoter activity in gadd153-silenced cells. We found that, silencing gadd153 expression results in a ∼50% reduction in the 27-OHC-induced increase in NF-κB transcriptional activity (Fig. 4f). Gadd153-silenced cells treated with 27-OHC exhibited a ∼1.7-fold increase in NF-κB transcriptional activity compared to a ∼3.5-fold increase in NF-κB transcriptional activity in native cells treated with 27-OHC (Fig. 4f). Dual-luciferase assay also demonstrated that knocking-down gadd153 expression in 27-OHC treated SH-SY5Y cells decreased the 27-OHC-induced increase in BACE1 promoter activity by ∼56% (Fig. 4g). Gadd153-silenced cells treated with 27-OHC exhibited a ∼2-fold increase in BACE1 promoter activity compared to a ∼4.2-fold increase in BACE1 promoter activity in native cells treated with 27-OHC (Fig. 4g). These data suggest that gadd153 expression is both necessary and mediates the 27-OHC-induced increase in BACE1 expression via NF-κB activation. However, the silencing of gadd153 expression did not alter the basal NF-κB transcription activity (Fig. 4f) and BACE1 promoter activity (Fig. 4g) as well as did not produce any effect on the extent of basal NF-κB binding to the BACE1 promoter region (Fig. 4e).

RETRACTED

Western blots for gadd153 show a strong band in hippocampus from the 3xTg-AD mice of 3, 6 and 12 months of age (Fig. 4h). NF-κB (p50) levels are highly detected in 6 and 12 month-old 3xTg-AD mice, but barely detected in the 3 month-old mice (Fig. h). BACE1 levels were substantially increased in the 12 month-old mice compared to 3 or 6 month-old mice. These results indicate that gadd153 protein levels are detected earlier than translocation of NFkB (p50) to the nucleus, which in turn precedes the increase in BACE1 levels. It is noteworthy to mention that Aβ levels increase the 3xTg-AD of more than 6 month of age [28].

As 27-OHC-induced increased expression of gadd153 increases BACE1 expression via NF-κB activation in human neuroblastoma SH-SY5Y cells, we investigated the involvement of gadd153 in 27-OHC-induced increase in Aβ production. Silencing of gadd153 expression effectuated a ∼33% reduction in the 27-OHC-induced increase in intracellular Aβ42 and a ∼22% decrease in 27-OHC-induced increase in intracellular Aβ40 (Fig. 5a,b). Intracellular Aβ42 levels were ∼1.3-fold the basal levels in gadd153-silenced cells treated with 27-OHC compared to ∼2-fold the basal levels in native cells treated with 27-OHC (Fig. 5a). Intracellular Aβ40 levels were not significantly different than the basal levels in gadd153-silenced cells treated with 27-OHC compared to ∼1.7-fold the basal levels in native cells treated with 27-OHC (Fig. 5b). Silencing of gadd153 expression also elicited ∼30% reduction in the 27-OHC-induced increase in secreted Aβ42 and ∼31% decrease in 27-OHC-induced increase in secreted Aβ40 (Fig. 5c,d). Secreted Aβ42 levels were ∼1.3-fold the basal levels in gadd153-silenced cells treated with 27-OHC compared to ∼1.9-fold the basal levels in native cells treated with 27-OHC (Fig. 5c). Similarly, secreted Aβ40 levels were ∼1.2-fold the basal levels in gadd153-silenced cells treated with 27-OHC compared to ∼1.8-fold the basal levels in native cells treated with 27-OHC (Fig. 5d). These data suggest the involvement of gadd153 in the 27-OHC-induced increase in Aβ. However, consistent with the lack of effect of the gadd153 siRNA on the basal expression levels of BACE1 and BACE1 promoter activity, the silencing of gadd153 expression did not elicit significant effects on the basal levels of Aβ42 (intracellular and secreted) and Aβ42 (intracellular and secreted) (Fig. 5a-d).

RETRACTED

**Figure 5:** Gadd153 expression is necessary for 27-OHC-induced increase in the levels of Aβ40 and Aβ42. (a,b) ELISA immunoassay demonstrates that siRNA to gadd153 expression attenuates the 27-OHC-induced increase in levels of intracellular and secreted Aβ42 and Aβ40. Data is expressed as Mean+S.E.M and includes determinations made in four separate cell culture experiments (n = 4). *p<0.05, **p<0.01, and ***p<0.001 versus control, ^††^ p<0.01 and ^†††^ p<0.001 versus 27-OHC.

### 27-OHC Increases the Activation of NF-κB via the Phosphorylation of IKK in gadd153-Dependent Manner

Next, we investigated the mechanism involved in the 27-OHC-induced gadd153-mediated increase in NF-κB activation. NF-κB activation is regulated by the IκBα (inhibitor of kappa B α) protein which masks the nuclear localization signal of the NF-κB subunits and sequesters the NF-κB complex sequestered in the cytosol [25], [26]. NF-κB activation entails the phosphorylation-evoked and proteasome-mediated degradation of IκB proteins resulting in the unmasking of the nuclear localization sequence of NF-κB heterodimeric [29], [30]. The IKK (IκB kinase) triad complex (composed of the catalytic subunits IKKα and IKKβ and the regulatory subunit IKKγ) activates NF-κB signaling pathway and allows the nuclear translocation of NF-κB heterodimeric complex by phosphorylation of the IκBα protein [30]–[32]. IKK complex is itself is activated by phosphorylation of Ser^176^ and Ser^180^ in the catalytic loop of IKKα and Ser^177^ and Ser^181^ in the catalytic loop of IKKβ [33]. Therefore, we determined the effects of 27-OHC on the phosphorylation of IKKα/β in the native and gadd153-deficient cells. We found that 27-OHC-evokes a 4.5-fold increase in phosphorylation of IKKα at Ser^176^/Ser^180^ and a 3-fold increase in the phosphorylation of IKKβ at Ser^177^/Ser^181^, thereby accounting for NF-κB activation (Fig. 6a,b). Interestingly, gadd153-silenced cells did not exhibit any increase in IKKα/β phosphorylation in response to 27-OHC, an effect consistent with the lack of NF-κB activation in gadd153-deficient cells treated with 27-OHC. We also found that while 27-OHC induces a significant decrease in IKBα levels and a significant increase in the phosphorylation of IKBα and β, siRNA to gadd153 reverses the 27-OHC-induced alterations in IKBα and p- IKBα levels (c,d). This data indicate that 27-OHC increases the degradation of IKBα.

**Figure 6:** 27-OHC increases the activation of NF-κB via the phosphorylation of IKKα/β which is dependent on gadd153 expression. 27-OHC induces a significant increase in the phosphorylation of IKKα/β, and siRNA to gadd153 reverses the 27-OHC-induced increase in phosphorylation of IKKα/β (a,b). 27-OHC induces a significant decrease in IKBα levels and a significant increase in the phosphorylation of IKBα; siRNA to gadd153 reverses the 27-OHC-induced alterations in IKBα and p- IKBα levels (c,d). Data is expressed as Mean+S.E.M and includes determinations made in four separate cell culture experiments (n = 4). ***p<0.001 versus control; ^††^ p<0.01 versus 27-OHC and ^†††^ p<0.001 versus 27-OHC.

RETRACTED

## Discussion

This study was conceived to elucidate signaling intermediates and transcription factors involved in the regulation of BACE1 expression. We determined the role of the ER stress-induced transcription factor gadd153 and the ubiquitous transcription factor NF-κB in the regulation of BACE1 expression levels in human neuroblastoma cells treated with the oxysterol 27-OHC. We demonstrate that 27-OHC induces BACE1 expression by increasing the activation and nuclear translocation of the transcription factor NF-κB in a gadd153-dependent manner. We found that silencing gadd153 expression significantly attenuated the 27-OHC-induced increase in NF-κB activation and NF-κB-mediated BACE1 expression. We further demonstrate that 27-OHC-induced increase in gadd153 expression results in the phosphorylation of IKKα/β and consequently activation in NF-κB and NF-κB mediated increase in BACE1 expression. Our data also shows gadd153 and NF-ΚB activation in the 3xTg-AD mice, suggesting that these transcription factors may contribute to the increase in BACE1 and the generation of Aβ peptide accumulation in these mice.

AD is a multifactorial disease with several factors likely contributing to its pathogenesis. Altered levels of sphingolipidome, ceramides, saturated fatty acids and several phospholipids may be involved in AD [34]–[39]. Previous studies from our laboratory have demonstrated that the cholesterol metabolite 27-OHC increases the expression levels of BACE1 and Aβ, and may also increase the risk for AD [16], [17], [40]. The aspartyl protease BACE1 catalyzes the rate-limiting step in the amyloidogenic processing of APP to generate the Aβ peptide [2], [3]. Some studies have found BACE1 expression levels to be increased in AD [6], [7], while other studies found no changes in BACE1 expression [41]–[43]. Preponderance of contemporary literature now overwhelmingly implicates increased BACE1 protein levels and activity in AD [4]; [44]–[46]. AD brains exhibit increased BACE1 protein levels and activity [4]; [6]; [44]. There is growing consensus that this increase in BACE1 plays a role in the neurodegenerative cascade that leads to AD. Interestingly, there is also suggestion that a positive feedback loop exists between amyloid plaques and BACE1 expression levels. Vassar and colleagues have recently demonstrated that BACE1 is up-regulated in neurons in the immediate vicinity juxtaposing the amyloid plaques [47]. Furthermore, the same study also demonstrated that BACE1 elevation in the neurons that surround the amyloid plaques is an early event preceding the subsequent neuronal loss that eventually occurs, thereby dispelling the speculation that the elevation in BACE1 levels and activity is an epiphenomenon that merely accompanies neuronal loss. Moreover, neuritic plaques containing a dense core of Aβ42 are able to elevate BACE1 expression levels in dystrophic neurites, but not diffuse plaques in transgenic mouse models [47]; [48]. The BACE1 transcription is modulated by a plethora of transcription factors and multitude of transcription factor binding sites have been found in the BACE1 promoter region including those for NF-κB, YY1, Sp1, and PPARγ among others [49]. In this study we determined the role of NF-κB in the 27-OHC-induced increase in BACE1 expression. To this end, we used sc514 to inhibit the activation of NF-κB in SH-SY5Y cells concomitantly treated with 27-OHC. We found that the NF-κB inhibitor significantly reduces the 27-OHC-induced increase in BACE1 expression levels. 27-OHC failed to evoke a similar magnitude of increase in BACE1 expression levels in cells concomitantly treated with sc514 compared to cells treated with 27-OHC alone. 27-OHC also induced the nuclear translocation of the p65 and the p50 NF-κB subunits. To further implicate the increased nuclear translocation of the p65 and the p50 NF-κB subunits with the increased expression of BACE1, we performed a ChIP assay to determine the binding of NF-κB to the BACE1 promoter region. Multiple studies have reported the modulation of BACE1 expression by NF-κB binding to the κB sites in the BACE1 promoter [12], [13]. Using ChIP analysis, we found that 27-OHC induced a marked increase in NF-κB binding to the BACE1 promoter region. To further demonstrate that the increase in the binding of NF-κB in the BACE1 promoter region does indeed result in the modulation of NF-κB-mediated BACE1 gene expression, we performed an NF-κB reporter activity assay to assess NF-κB transcriptional activity and a BACE1 promoter assay to assess changes in BACE1 gene transcription. We found that 27-OHC substantially increases NF-κB reporter activity and BACE1 promoter activity. Furthermore, the NF-κB inhibitor attenuated the 27-OHC-induced increase in BACE1 promoter activity thereby further implicating NF-κB in the 27-OHC-induced upregulation of BACE1 expression. Indeed, NF-κB activity has been found to be increased in autopsied AD-brain tissue as well as increased NF-κB immunoreactivity has been observed in proximity to amyloid plaques [12], [13], [50], [51]. As BACE1 catalyzes the rate-limiting step in the genesis of Aβ peptide via the amyloidogenic processing of APP and given that BACE1 expression levels are tightly associated with Aβ levels, we determined the effects of the NF-κB inhibitor sc514 on the 27-OHC-induced increase in Aβ levels. The NF-κB inhibitor significantly mitigated the 27-OHC-induced increase in both intracellular as well as secreted forms Aβ42 and Aβ40.

RETRACTED

The ER is an organelle of fundamental importance to cell functions as it is the Ca^2+^ storage site and where surface and secreted proteins are synthesized, folded and assembled before being transported. Mounting evidence indicates a role of ER stress in the pathophysiology of many diseases including AD [8]–[10]. ER dyshomeostasis triggers stress signaling by activating the unfolded protein response (UPR) [52]. The UPR signaling is intended to protect cells from the consequences of changes in Ca^2+^ levels and the buildup of misfolded proteins. However, intense or sustained ER stress activates deleterious cascades including the activation of the transcription factor gadd153. It is significant how gadd153 activation is linked to AD as this transcription factor regulates genes and proteins related to the pathophysiology of this disease (see for review [10]). It is also significant that PS1 mutations, a risk factor for familial AD, increases gadd153 protein translation [53]. Previous studies from our laboratory have demonstrated that the ER stress-induced transcription factor gadd153 mediates the 27-OHC-induced increase in BACE1 expression in hippocampal organotypic slices from adult rabbits [40]. However, the molecular mechanisms and signal transductional intermediates utilized by gadd153 to elicit an increase in BACE1 expression had not been determined prior to this study. BACE1 expression is markedly induced by cellular stressors such as oxidative stress [54], hypoxia [55], [56] and glucose deprivation [57] as well as aging [58]. Interestingly, gadd153 expression is also induced by the same cellular stressors and glucose and nutrient deprivation [52]. It is therefore conceivable that gadd153 could be a key factor instigating this stress-mediated induction of BACE1 expression.

Recent emerging evidence has implicated ER stress-induced gadd153 expression in NF-κB activation [11]. Therefore, we determined the role of NF-κB in 27-OHC-induced gadd153-mediated upregulation of BACE1. To this end, we knocked-down the expression of gadd153 via siRNA-mediated gene silencing and determined the effects on basal NF-κB levels as well as 27-OHC-induced increased NF-κB levels in the nuclear homogenates. Silencing gadd153 expression did not affect the basal levels of p65 and p50 NF-κB subunits in the nucleus. However, gadd153 silencing reversed the 27-OHC-induced increase in p65 and p50 NF-κB levels in the nucleus. This suggests that increased expression of gadd153 mediates the 27-OHC-induced activation and nuclear translocation of p65 and p50 NF-κB. Consistent with our previous study in hippocampal organotypic slices from adult rabbits [40], silencing of gadd153 expression significantly mitigated the 27-OHC-induced increase in BACE1 expression without affecting the basal expression of BACE1. To further implicate NF-κB as the intermediate in 27-OHC-induced gadd153-mediate increase in BACE1 expression, we subsequently performed EMSA and ChIP analyses to study the binding of NF-κB to the BACE1 promoter region in response to treatment with 27-OHC in a gadd153-deficient paradigm. Consistent with the observation of lack of commensurate increase in BACE1 expression in gadd153-silenced cells treated with 27-OHC, silencing gadd153 expression significantly attenuated the binding of NF-κB in the BACE1 promoter region as revealed by EMSA and ChIP analysis. However, changes in NF-κB binding to the BACE1 promoter may not necessarily evoke changes in transcription of BACE1. Therefore, we next performed NF-κB reporter activity assay to assess NF-κB transcriptional activity and also BACE1 promoter analysis to assess BACE1 transcriptional changes in gadd153-silenced cells treated with 27-OHC. Silencing gadd153 expression significantly reduced the 27-OHC-induced increase in NF-κB reporter activity and BACE1 promoter activity, thereby suggesting that gadd153 mediates the 27-OHC-induced increase in NF-κB transcriptional activity and BACE1 transcription. Our data is consistent with the observation that many signal transduction pathways that are actuated by cellular stressors that evoke ER stress do also indeed increase BACE1 expression levels. However, no gadd153 binding sites have been identified yet in the BACE1 promoter suggesting that gadd153 may not directly regulate BACE1 expression. Recently, it was demonstrated that ER stress-induced activation of gadd153 increases NF-κB signaling [11]. We explored the possibility of this gadd153-NF-κB crosstalk as 27-OHC induces the expression of gadd153 as well as NF-κB activation. Indeed, we found that increased gadd153 expression by 27-OHC positively regulates NF-κB activation and expression of NF-κB target genes. Specifically, we found that 27-OHC induced phosphorylation of IKKα/β that results in the phosphorylation and proteasomal degradation of IκB proteins culminating in the activation of NF-κB is regulated positively by gadd153. However, further studies are warranted to examine the signaling intermediates involved in the gadd153- NF-κB crosstalk that regulates BACE1 expression and therefore could represent a potential therapeutic target in AD.

RETRACTED

In summary, we demonstrate that the ER stress-activated transcription factor gadd153 positively regulates BACE1 expression via the activation of NF-κB signaling cascade (Fig. 7). Our study provides a valuable insight into the putative molecular mechanisms and signal transduction cascades that regulate BACE1 expression and is therefore of high relevance to the search and design of therapeutic intervention that can reduce BACE1 as well as Aβ overproduction, and AD progression.

**Figure 7:** Schematic representation of the molecular mechanisms involved in the 27-OHC-induced increase in BACE1 expression. 27-OHC activates gadd153 (1) which evokes the phosphorylation of the IKK-complex (2). Phosphorylation IKK complex (3) results in the phosphorylation and subsequent proteasomal degradation of IκB (4), thereby releasing the p65-p50 NF-κB dimer from inhibitory sequestration in the cytosol and allowing the p65-p50 NF-κB dimer to translocate to the nucleus (5). The translocated p65-p50 NF-κB dimer binds to distinct κB sites in the BACE1 promoter region and upregulates BACE1 expression (5). Increased gadd153 expression by 27-OHC may also induce NF-κB activation, nuclear translocation, and subsequently increase BACE1 expression by other mechanism that are yet to be elucidated (6). siRNA to gadd153 reduces the 27-OHC-induced nuclear translocation of NF-κB and thereby attenuates the increase in BACE1(7). The NF-κB inhibitor sc514 also decreases the 27-OHC-induced increase in BACE1 expression by inhibiting the nuclear translocation of NF-κB and subsequent increase in NF-κB-mediated transcription of BACE1 (8).
